The article "LDH and GGT/ALT Ratio as Novel Prognostic Biomarkers in Hepatocellular Carcinoma Patients after Liver Transplantation" was retracted in 2023. Reasons: signs of a paper mill; compromised peer review; unreliable results or conclusions.

# LDH and GGT/ALT Ratio as Novel Prognostic Biomarkers in Hepatocellular Carcinoma Patients after Liver Transplantation

**DOI:** 10.1155/2021/9809990

**Published:** 2021-11-20

**Authors:** Qi Zhang, Xingyuan Jiao

**Affiliations:** Organ Transplant Center, The First Affiliated Hospital, Sun Yat-sen University, Guangzhou, China

## Abstract

**Background:**

Liver inflammation indices reflect its inflammatory microenvironment, which may play a role in the proliferation, invasion, and migration of carcinoma. This study is aimed at exploring the prognostic significance of serum lactate dehydrogenase (LDH) levels and gamma-glutamyl transferase (GGT)/alanine aminotransferase (ALT) ratio in hepatocellular carcinoma after liver transplant (LT).

**Methods:**

We retrospectively analyzed data from 155 patients with a pathologically confirmed diagnosis of hepatocellular carcinoma who received LT between January 2013 and September 2017. We used receiver operating characteristics (ROC) curves to determine the optimal LDH and GGT/ALT ratio cut-off values. The Kaplan–Meier method and the logarithmic rank test were used to compare the survival curves without recurrence (RFS) and overall survival (OS). Univariate and multivariate analyses were used to identify factors associated with survival.

**Results:**

Serum LDH levels were significantly associated with the Child-Pugh score (*P* = 0.037), largest tumor size (<50 vs. ≥50 mm) (*P* = 0.017), tumor count (<3 vs. ≥3) (*P* = 0.009), microvascular invasion (*P* = 0.006), and the Milan criteria (*P* ≤ 0.001). The serum GGT/ALT ratio was significantly correlated with alpha-fetoprotein (AFP) levels (of <400 vs. ≥400 ng/ml) (*P* ≤ 0.001), largest tumor size (of <50 vs. ≥50 mm) (*P* ≤ 0.001), the Edmondson grade (I-II vs. III-IV) (*P* = 0.028), microvascular invasion (*P* ≤ 0.001), and the Milan (*P* = 0.002) and Hangzhou criteria (*P* = 0.018). The survival curves showed that the patients with high LDH and the GGT/ALT ratio were associated with poor RFS and OS (*P* < 0.05). Univariate and multivariate analyses showed that AFP levels of ≥400 ng/ml, largest tumor size of ≥50 mm, microvascular invasion, LDH levels of ≥213.5 U/l, and the GGT/ALT ratio of ≥3.1338 were factors independently associated with RFS.

**Conclusion:**

Elevated LDH levels and the GGT/ALT ratio before LT were associated with poor OS and RFS in the present study. These factors could be used in the prognostication of patients with hepatocellular carcinoma undergoing LT.

## 1. Introduction

Hepatocellular carcinoma (HCC) is the most common form of primary liver tumor and is one of the leading causes of cancer-related deaths worldwide [1, 2]. Its incidence and associated mortality continue to increase and attract attention. HCC is associated with several risk factors, such as hepatitis B virus and hepatitis C virus (HCV) infections, which account for most HCC cases, in particular those diagnosed in East Asia [3]. Furthermore, HCC has also been associated with aflatoxin exposure, heavy alcohol intake, obesity, smoking, and type 2 diabetes [4, 5].

The article "LDH and GGT/ALT Ratio as Novel Prognostic Biomarkers in Hepatocellular Carcinoma Patients after Liver Transplantation" was retracted in 2023. Reasons: signs of a paper mill; compromised peer review; unreliable results or conclusions.

Current treatments for HCC include surgical resection, liver transplant (LT), transcatheter arterial chemoembolization (TACE), and radiofrequency ablation (RFA) [6]. LT is currently considered the most definitive treatment option for HCC, as it removes the tumor as well as the unhealthy organ, which, when retained, remains at risk of HCC recurrence due to the presence of cirrhotic tissue [7]. Patient prognosis following LT is associated with the risk of HCC recurrence; thus, several selection criteria have been established to help select patients most likely to benefit from an LT, including the Milan criteria (the diameter of a single tumor was less than 5 cm, and the maximum diameter of multiple tumors was less than 3 cm) and the Hangzhou criteria (tumor diameter < 8 cm or tumor diameter > 8 cm, and preoperative AFP < 400 ng/ml and tumor histological grade were high and medium differentiation). Although we can apply these strict criteria to clinical trials, 5-year recurrence-free survival (RFS) of HCC after LT is only 75% [8].

In the clinical setting, abdominal ultrasound, computed tomography, magnetic resonance imaging, and alpha-fetoprotein (AFP) level assessments are commonly used to estimate the risk of HCC recurrence after surgery. These results sometimes can only work when there is a definite recurrence of HCC, so we want to seek some indices which can predict the survival of HCC after LT easily. Recent studies have shown that tumor inflammatory microenvironments can contribute to the risk of proliferation, invasion, and migration of carcinoma [9], suggesting the role of preoperative peripheral blood inflammation markers, such as C-reactive protein levels [10], platelet-to-lymphocyte ratio [11], and neutrophil-to-lymphocyte ratio [12, 13] in the postoperative period. In addition, liver inflammation indices such as gamma-glutamyl transferase (GGT), alanine aminotransferase (ALT), aspartate aminotransferase, and lactate dehydrogenase (LDH) levels have been associated with the risk of HCC recurrence after hepatectomy [14, 15]. Notwithstanding, there have been few studies on the relationship between liver inflammation indices and HCC prognosis after LT. The present study is aimed at examining the prognostic value of LDH levels and the GGT/ALT ratio in patients with HCC who underwent LT while adjusting for clinicopathological characteristics.

The article "LDH and GGT/ALT Ratio as Novel Prognostic Biomarkers in Hepatocellular Carcinoma Patients after Liver Transplantation" was retracted in 2023. Reasons: signs of a paper mill; compromised peer review; unreliable results or conclusions.

## 2. Methods

### 2.1. Ethics

This study was performed according to the principles of the Declaration of Helsinki and approved by the Ethics Committee of the First Affiliated Hospital of Sun Yat-sen University. All transplanted organs came from legal donors. Before the LT, each recipient provided informed consent to their data being used for research purposes.

### 2.2. Patients

We retrospectively analyzed the clinical records of 155 patients that were diagnosed with HCC and received an LT at the First Affiliated Hospital of Sun Yat-sen University between January 2013 and September 2017; these patients were followed up until October 2020. Data were extracted from the China Liver Transplantation Register (http://www.cltr.org/) and patient medical records; the variables of interest included recipient age, sex, height and weight, liver encephalopathy status, ascites, pretransplant treatments, and preoperative laboratory findings, including total bilirubin and albumin levels, prothrombin time, international normalized ratio value, and GGT, ALT, LDH, creatinine, and AFP levels. We determined the number and size of tumors and the macrovascular invasion status based on imaging findings. The Edmondson tumor grade (the main methods of pathological classification of HCC at present) and microvascular invasion status were determined based on pathological findings. We also calculated body mass index, model for end-stage liver disease (MELD) score, and the Child-Pugh class and GGT/ALT ratio. All patients survived for at least 45 days postoperatively; there was no case of surgery-related death in this cohort.

### 2.3. Inclusion and Exclusion Criteria

Patients were eligible for this study if they met the following criteria: (1) histologically confirmed HCC, (2) absence of distant metastases, and (3) age 18-75 years. Patients were excluded from this study if they met any of the following criteria: (1) perioperative death within 45 days, (2) incomplete clinical and follow-up information, (3) combined with other cancers, (4) diagnosis of comorbidities, (5) need for repeat transplantation, or (6) multiple organ transplantation.

### 2.4. Treatment and Follow-Up

Some patients received several treatments prior to LT, for example, surgical resection, TACE, and RFA. In such cases, we assessed imaging findings to confirm that indications for LT were present. For all patients, survival status was determined after a minimum of 3 years of follow-up. Patients were contacted by phone or in person. The follow-up data included the date of HCC recurrence or death as well as the cause of death. All recipients were followed up regularly; peripheral blood and imaging findings were used to assess HCC recurrence; patients that required hospitalization were admitted for further treatment.

The article "LDH and GGT/ALT Ratio as Novel Prognostic Biomarkers in Hepatocellular Carcinoma Patients after Liver Transplantation" was retracted in 2023. Reasons: signs of a paper mill; compromised peer review; unreliable results or conclusions.

### 2.5. Statistical Analysis

All data were presented as counts (%) or medians (IQR). Continuous variables were compared using the *t*-test; categorical variables were compared using the chi-square test. Receiver operating characteristic curve (ROC) analysis and the highest Youden index value (sensitivity + specificity − 1) were used to determine the optimal cut-off value of LDH levels and the GGT/ALT ratio. The Kaplan–Meier method and the log-rank test were used to compare RFS and OS curves. Multivariate and univariate Cox regression analyses were performed to obtain a risk model. All statistical analyses were performed using SPSS version 23.0 (SPSS, Chicago, IL, USA). The *P* values of <0.05 were considered indicative of a statistically significant finding.

## 3. Results

### 3.1. Clinical Characteristics of Patients

The patient's clinical characteristics are presented in Table 1. A total of 155 patients were enrolled in this study, including 142 (91.6%) and 13 (8.3%) men and women, respectively, with an overall median age of 50 (range, 42-58) years. According to the Child-Pugh class system, 47 (30.3%), 87 (56.1%), and 21 (13.5%) patients were classified as Classes A, B, and C, respectively. The median MELD score of these patients was 11 (8-18) points. Before LT, 30 (19.3%), 74 (47.7%), and 29 (18.7%) patients received surgical resection, TACE, and RFA, respectively. Some patients received multiple pre-LT treatments. The Edmondson pathological grades of I-II and III-IV were observed in 111 (71.6%) and 44 (28.4%) patients, respectively. A total of 121 (78.1%) and 115 (74.2%) patients had macrovascular and microvascular invasion, respectively. The median largest tumor size was 11 mm (range, 8-18). A total of 110 (71.0%) and 49 (31.6%) patients met the Hangzhou and Milan criteria, respectively. HCC recurrence was observed in 65 (41.9%) patients.

### 3.2. Cutoff Values for LDH Levels and the GGT/ALT Relationship

The analysis of the ROC curve and the Youden index revealed that the optimal cutoff values of LDH levels and the GGT/ALT ratio to predict the recurrence of HCC after surgery were 80.5 U/l (AUC = 0.647, *P* = 0.002) and 3.1338 (AUC = 0.744, *P* = 0.001), respectively (Figure 1 and Table 2).

### 3.3. LDH Levels, the GGT/ALT Ratio, and Other Clinicopathological Features

Serum LDH levels were significantly associated with the Child-Pugh class (*P* = 0.037), largest tumor size (<50 vs. ≥50 mm) (*P* = 0.017), tumor number (3 vs. 3) (*P* = 0.009), microvascular invasion (*P* = 0.006), and Milan criteria (*P* = 0.001). Serum ratio of GGT/ALT was significantly associated with AFP levels (<400 vs. ≥400 ng/ml) (*P* ≤ 0.001), largest tumor size (<50 vs. ≥50 mm) (*P* = 0.001), Edmondson grade (I-II vs. III-IV) (*P* = 0.028), microvascular invasion status (*P* = 0.001), and the Milan (*P* = 0.002) and Hangzhou criteria (*P* = 0.018) (Table 3).

The article "LDH and GGT/ALT Ratio as Novel Prognostic Biomarkers in Hepatocellular Carcinoma Patients after Liver Transplantation" was retracted in 2023. Reasons: signs of a paper mill; compromised peer review; unreliable results or conclusions.

### 3.4. Kaplan–Meier Survival Curves of each Patient Group

The RFS and OS curves for patients in the high and low LDH level groups and in the high and low GGT/ALT ratio groups are presented in Figures 2(a)–2(d), respectively. The high level of LDH and the GGT/ALT ratio was significantly associated with poor RFS (P = 0.001 and P = 0.001) and poor OS (P = 0.008 and P = 0.001, respectively).

### 3.5. Risk Factors Associated with the Prognosis of HCC

RFS was used at the outcome representative of patient prognosis, as OS may be affected by a wider range of factors. Univariate analyses revealed that AFP levels of ≥400 ng/ml, largest tumor size of 50 mm, Edmondson grade IIIIII-IV, microvascular invasion, LDH levels of ≥213.5 U/L, and the GGT/ALT ratio of 3.1338 were significantly associated with poor RFS (Table 4). Multivariate analysis revealed that AFP levels of ≥400 ng/ml, largest tumor size of ≥50 mm, microvascular invasion, LDH levels of ≥213.5 U/L, and the GGT/ALT ratio of ≥3.1338 were independent risk factors for RFS (Table 4).

## 4. Discussion

The prognosis of HCC remains a major focus of research. Currently, LT is considered the most effective treatment for HCC worldwide. Any type of treatment is aimed at reducing the risk of HCC recurrence. The Milan criteria are the LT eligibility criteria associated with excellent long-term outcomes [16]. However, approximately 30% of patients who meet this criterion experience post-LT recurrence [17]. Risk factors associated with post-LT outcomes in HCC patients have previously been reported and include histological grade, vascular invasion status, and number and diameter of nodules [18, 19]. However, these factors are difficult to assess before an LT; therefore, serum-based biomarkers that can be easily obtained before surgery have become the focus of research in recent years.

GGT is a membrane-bound enzyme that plays a crucial role in glutathione (GSH) metabolism, specifically in the degradation of extracellular GSH by cleaving its gamma-glutamyl bond [20] and promoting the recovery of amino acids for intracellular glutathione synthesis [21]. GSH is the main water-soluble antioxidant within the cell, while GGT is involved in a defense mechanism against oxidative stress [22]; consequently, high levels of GGT are indicative of oxidative stress within cells, which, in turn, can participate in tumorigenesis [23]. A growing body of evidence suggests that elevated serum GGT levels in patients with HCC may be a prognostic marker [15, 24]. ALT levels are often used to evaluate hepatocyte damage; ALT can be released from damaged hepatocytes into the blood. In acute and chronic viral hepatitis, alcoholic hepatitis, and cirrhosis, ALT levels are elevated to varying degrees; meanwhile, in patients with HCC, ALT levels tend to be within or below the normal range [25]. Based on these findings, we hypothesized that the GGT/ALT ratio may reflect the invasiveness of HCC. This index was used for the first time to evaluate the effect of antiviral therapy in patients with chronic HCV [26]. Ju et al. reported that the preoperative serum GGT/ALT ratio was associated with Child-Pugh class A HCC [14]. To the best of our knowledge, the present study is the first to use this index in the evaluation of HCC prognosis post-LT. Moreover, this study offered evidence to confirm our hypothesis: we conclude that the preoperative GGT/ALT ratio of ≥3.1338 is associated with a reduced RFS (*P* < 0.05) and OS (*P* < 0.05). Other factors associated with reduced survival include higher AFP levels (*P* = 0.001), larger tumor size (*P* ≤ 0.001), higher Edmondson grade (*P* = 0.028), and the presence of microvascular invasion (*P* = 0.001), all of which suggest that the GGT/ALT ratio is correlated with the degree of HCC malignancy. Multivariate analysis revealed that the GGT/ALT ratio of 3.1338 was an independent prognostic factor for RFS. The present findings suggest that the GGT/ALT ratio may be clinically useful in the prognosis of patients with HCC.

The article "LDH and GGT/ALT Ratio as Novel Prognostic Biomarkers in Hepatocellular Carcinoma Patients after Liver Transplantation" was retracted in 2023. Reasons: signs of a paper mill; compromised peer review; unreliable results or conclusions.

LDH levels are assessed during routine preoperative checks. LDH is a critical metabolic enzyme that converts pyruvate to lactate under anaerobic conditions. A growing body of evidence suggests that abnormal LDH levels are associated with increased rates of tumor metastasis and recurrence, as well as poor treatment outcomes in several cancer types [27, 28], including HCC [29]. In the present study, elevated LDH levels (≥213.5 U/l) were significantly associated with a higher Child-Pugh class (*P* = 0.037), largest tumor size of ≥50 mm (*P* = 0.017), tumor count of ≥3 (*P* = 0.009), and microvascular invasion (*P* = 0.006); these findings are consistent with those of previous studies. Furthermore, LDH levels were associated with post-LT RFS in patients with HCC.

Previous studies have examined the contribution of LDH to tumor progression. Low oxygen levels (hypoxia) characterize cancer cells and influence their function. In addition, hypoxia is an important component of the tumor microenvironment (TME) as it alters the extracellular matrix, modulates the immune response of the tumor, and increases the rate of angiogenesis [30]. Under these conditions, LDH can play a significant role in the energy supply of carcinoma cells. Even in the presence of oxygen, a phenomenon called the Warburg effect refers to carcinoma cells that preferentially convert glucose to lactate in aerobic glycolysis [31]. Changes in metabolic pathways can contribute to tumor proliferation and growth by ensuring energy and substrate supply. These alterations could create advantageous reducing conditions in the TME that are optimal for cancer survival [32]. Elevated LDH levels are common in the malignant progression of carcinoma, including HCC.

The article "LDH and GGT/ALT Ratio as Novel Prognostic Biomarkers in Hepatocellular Carcinoma Patients after Liver Transplantation" was retracted in 2023. Reasons: signs of a paper mill; compromised peer review; unreliable results or conclusions.

Finally, multivariate analysis demonstrated that AFP levels (400 ng/ml), the largest tumor size (50 mm), and microvascular invasion were independently associated with RFS. These factors were recognized in the development of HCC, so we would not discuss them here.

This study has several limitations. Since this study was retrospective and single-centered, the sample size was small and may have yielded biased estimates. Future multicenter and prospective studies with large sample sizes are required to confirm our findings.

## 5. Conclusions

Elevated pre-LT LDH levels and GGT/ALT ratio are associated with poor OS and RFS and may be clinically useful in the prognostication of patients with HCC undergoing LT.

## Figures and Tables

**Figure 1:** Receiver operating characteristic curves for serum LDH levels (a) and the GGT/ALT ratio (b) in patients with hepatocellular carcinoma after a liver transplant. LDH: lactate dehydrogenase; GGT: gamma-glutamyl transferase; ALT: alanine aminotransferase.

**Figure 2:** Relationship between LDH levels (a, b) and the GGT/ALT ratio (c, d), and overall survival without recurrence. LDH: lactate dehydrogenase; GGT: gamma-glutamyl transferase; ALT: alanine aminotransferase.

**Table 1:** Clinical characteristics of patients.

Characteristics	Median (25th-75th percentile) or no. (%)
Sex	
Male	142 (91.6)
Female	13 (8.3)
Age (years)	50 (42-58)
Child-Pugh class	
A	47 (30.3)
B	87 (56.1)
C	21 (13.5)
MELD score	11 (8-18)
Tumor number	
<3	82 (52.9)
≥3	73 (47.1)
Largest tumor size (mm)	44 (25-80)
Edmondson grading	
I-II	111 (71.6)
III-IV	44 (28.4)
AFP (ng/ml)	117.24 (10.12-2614.33)
BMI (kg/m^2^)	22.15 (20.42-24.09)
Macrovascular invasion	
Yes	121 (78.1)
No	34 (21.9)
Microvascular invasion	
Yes	115 (74.2)
No	40 (25.8)
Pre-LT treatment	
Surgical resection	30 (19.3)
TACE	174 (47.7)
RFA	29 (18.7)
Milan criteria	
Yes	49 (31.6)
No	106 (68.4)
Hangzhou criteria	
Yes	110 (71.0)
No	45 (29.0)
HCC recurrence	65 (41.9)
Follow-up (months)	40 (22-54)
GGT (U/l)	111 (51-201)
ALT (U/l)	38 (25-58)
LDH (U/l)	208 (181-268)

The article "LDH and GGT/ALT Ratio as Novel Prognostic Biomarkers in Hepatocellular Carcinoma Patients after Liver Transplantation" was retracted in 2023. Reasons: signs of a paper mill; compromised peer review; unreliable results or conclusions.

**Table 2:** Comparisons of the Areas Under the Curve (AUC) values and the determination of the cut-off values.

	AUC	Cut-off	SE	95% CI	*P*
LDH	0.647	213.5	0.045	0.559-0.735	0.002
GGT/ALT	0.704	3.1338	0.042	0.621-0.787	0.000

**Table 3:** Relationship between LDH and GGT/ALT with clinicopathologic parameters.

Patient-related factors	LDH (U/l)		*P* value	GGT/ALT		*P* value
	<213.5	≥213.5		<3.1338	≥3.1338	
	*n* = 83	*n* = 72		*n* = 85	*n* = 70	
Sex			0.546			0.276
Male	75	67		76	66	
Female	8	5		9	4	
Age (years)			0.430			0.159
<60	65	60		72	53	
≥60	18	12		13	17	
Child-Pugh class			0.037			0.754
A	27	20		24	23	
B	40	47		50	37	
C	16	5		11	10	
Pre-LT treatment			0.458			0.719
Yes	51	40		51	40	
No	32	32		34	30	
AFP (ng/ml)			0.062			0.000
<400	56	38		63	31	
≥400	27	34		22	39	
Largest tumor size (mm)			0.017			0.000
<50	56	35		63	28	
≥50	27	37		22	42	
Tumor number			0.009			0.051
<3	52	30		51	31	
≥3	31	42		34	39	
Edmondson grading			0.841			0.028
I-II	60	51		67	44	
III-IV	23	21		18	26	
Macro-vascular invasion			0.936			0.521
Yes	18	16		17	17	
No	65	56		68	53	
Micro-vascular invasion			0.006			0.001
Yes	14	26		13	27	
No	69	46		72	43	
Milan criteria			0.001			0.002
Yes	36	13		36	13	
No	47	59		49	57	
Hangzhou criteria			0.973			0.018
Yes	59	51		67	43	
No	24	21		18	27	

**Table 4:** Univariate and multivariate analyses of factors for prediction of recurrence-free survival.

Characteristics	Univariate analysis			Multivariate analysis		
	HR	95% CI	*P* value	HR	95% CI	*P* value
Sex (male/female)	1.224	0.491-3.051	0.664			
Age (<60/≥60) (years)	0.904	0.483-1.693	0.753			
Child-Pugh stage (A/B/C)	1.118	0.757-1.652	0.574			
MELD score	1.017	0.993-1.041	0.179			
BMI (kg/m^2^)	0.970	0.896-1.051	0.459			
Tumor number (<3/≥3)	1.437	0.882-2.341	0.146			
Largest tumor size (<50/≥50) (mm)	2.795	1.701-4.593	0.000	1.841	1.096-3.091	0.021
Edmondson grading (I-II/III-IV)	1.805	1.081-3.015	0.024			0.279
Pre-LT treatment (yes/no)	1.077	0.653-1.776	0.770			
AFP (<400/≥400) (ng/ml)	3.320	2.017-5.466	0.000	2.120	1.260-3.568	0.005
Macrovascular invasion (yes/no)	1.639	0.929-2.892	0.088			
Microvascular invasion (yes/no)	2.863	1.729-4.742	0.000	1.771	1.043-3.010	0.035
GGT/ALT (<3.1338/≥3.1338)	3.361	1.998-5.654	0.000	2.008	1.208-3.609	0.008
LDH (<213.5/≥213.5) (U/l)	2.408	1.459-3.974	0.001	1.791	1.075-2.985	0.025

## Data Availability

The data used to support this study are available from the corresponding author upon request.
